# Severe Chromoblastomycosis-Like Cutaneous Infection Caused by *Chrysosporium keratinophilum*

**DOI:** 10.3389/fmicb.2017.00083

**Published:** 2017-01-25

**Authors:** Juhaer Mijiti, Bo Pan, Sybren de Hoog, Yoshikazu Horie, Tetsuhiro Matsuzawa, Yilixiati Yilifan, Yong Liu, Parida Abliz, Weihua Pan, Danqi Deng, Yun Guo, Peiliang Zhang, Wanqing Liao, Shuwen Deng

**Affiliations:** ^1^Department of Dermatology, People’s Hospital of Xinjiang Uygur Autonomous RegionUrumqi, China; ^2^Department of Dermatology, Shanghai Changzheng Hospital, Second Military Medical UniversityShanghai, China; ^3^Key Laboratory of Molecular Medical Mycology, Shanghai Changzheng Hospital, Second Military Medical UniversityShanghai, China; ^4^CBS-KNAW Fungal Biodiversity Centre, Royal Netherlands Academy of Arts and SciencesUtrecht, Netherlands; ^5^Medical Mycology Research Center, Chiba UniversityChiba, Japan; ^6^Department of Nutrition Science, University of NagasakiNagasaki, Japan; ^7^Department of Dermatology, First Hospital of Xinjiang Medical UniversityUrumqi, China; ^8^Department of Dermatology, The Second Affiliated Hospital of Kunming Medical UniversityKunming, China

**Keywords:** *Chrysosporium keratinophilum*, cutaneous infection, fungal infection, diagnosis, treatment

## Abstract

*Chrysosporium* species are saprophytic filamentous fungi commonly found in the soil, dung, and animal fur. Subcutaneous infection caused by this organism is rare in humans. We report a case of subcutaneous fungal infection caused by *Chrysosporium keratinophilum* in a 38-year-old woman. The patient presented with severe chromoblastomycosis-like lesions on the left side of the jaw and neck for 6 years. She also got tinea corporis on her trunk since she was 10 years old. *Chrysosporium keratinophilum* was isolated from the tissue on the neck and scales on the trunk, respectively. The patient showed satisfactory response to itraconazole therapy, although she discontinued the follow-up.

## Introduction

*Chrysosporium* species are saprophytic filamentous fungi occurring in soil, dung, animal fur, and bird feathers (Hocquette et al., 2005). *Chrysosporium keratinophilum* may cause mild infections in humans and is sometimes responsible for onychomycosis (Hocquette et al., 2005). However, subcutaneous infection resulting from *C. keratinophilum* has never been reported. Here, we present a case of severe chromoblastomycosis-like subcutaneous infection caused by *C. keratinophilum* from China.

## Case Report

A 38-year-old woman presented with a 4-year history of multiple verrucous nodules with a cauliflower-like appearance on her neck and face. The lesions were pruritic and progressively spread. Physical examination showed numerous verrucous nodules with superficial ulceration on the left side of her jaw and neck (**Figure 1A**). An isolated erythematous plaque with scale was also noted on her back (**Figure 1B**). The patient did not suffer from any known underlying disease or immunodeficiency. She noticed a first small nodule on her left ear without any trauma in 2010. The lesion gradually expanded to the left side of her neck. She did not pay attention to it until her pregnancy in 2012 when the lesions spread aggressively to the entire left side of the neck. Then she was admitted to our hospital. She had a history of tinea corporis when she was 10 years old; at that time, other family members had the similar problem. Because of the patient’s poor compliance with antifungal treatment (oral griseofulvin), the lesions on her trunk did not totally disappear but remained for years, although her family members were cured completely with the same therapy. Potassium hydroxide (KOH) direct examination of exudates from the plaque lesion in the neck and scales lesion from trunk revealed septate hyphal elements. Microscopic features of organisms from the two sites (her neck and trunk) were similar (**Figures 1C,D**). A biopsy taken from the lesion on the neck showed suppurative granulomata formation, and septate hyphal elements were found in the dermis and pus upon PAS (Periodic Acid-Schiff) staining (**Figures 2A,B**). Acid-fast staining was negative. Routine laboratory tests were unremarkable. Based on the histopathological and microscopic examination, a provisional diagnosis of a fungal infection was made, but no treatment was given during her pregnancy until her delivery when she received oral itraconazole (200 mg twice daily, BID) for 3 months. The rash dramatically reduced, and scaling lesions on her truck disappeared. However, the patient discontinued medication and was lost for follow-up. After 2 years (in 2014), the patient readmitted to our hospital with aggravated lesions on her neck again (**Figure 3A**). Scaling lesions were noticed on her trunk as well (**Figure 3B**). Therapy was given with itraconazole (200 mg, BID) for another 4 months. Plaques and nodules gradually became flat with scarring left (**Figure 3C**). The scaling lesions on her trunk had disappeared completely. Unfortunately, the patient was lost for follow-up again.

**FIGURE 1:** **(A)** Initial presentation: plaques and multiple verrucous nodules as a cauliflower-like appearance, superficial ulceration filled with pus on her left side of jaw and neck. **(B)** Scaling lesions spontaneously appeared on her trunk. **(C,D)** Direct examination of 10% Potassium hydroxide (KOH) wet mounts of exudates from surface plaque of neck and scales from the trunk revealed hyphae fractions (×400).

**FIGURE 2:** **(A,B)** Septate hyphae were present in the dermis. (PAS stain, ×100 and ×400).

**FIGURE 3:** **(A)** Aggravated lesion re-appeared on her neck. **(B)** Scaling lesions were also noticed on her trunk (arrows). **(C)** Lesions gradually disappeared after treatment.

## Mycology

Direct microscopy of exudates from the lesion on the neck and scales on the trunk revealed septate hyphal elements (**Figures 1C,D**). Both clinical specimens were cultured on potato dextrose agar (PDA) at 25°C for up to 2 weeks. Colonies grew slowly, appeared yellowish white, fluffy, with a dense, powdery center (**Figure 4A**). Microscopy of hyphal colonies revealed the same morphology, hyaline hyphae bearing conidia which were terminal or lateral, sessile or on short, cylindrical protrusions, thick-walled, obovoid to clavate with conspicuous basal scars (**Figure 4B**), which were phenotypically identified as a *Chrysosporium* species. The identification was further confirmed by sequencing of ITS region of rDNA using the Blast program in GenBank which yielded a 99% identity match with the strain IFM 55159 of *C. keratinophilum* (accession no. AB361655). The isolate from neck was deposited in the collection of the Centraalbureau voor Schimmelcultures Fungal Biodiversity Centre (CBS) under strain number 142081 and the IFM collection (Medical Mycology Research Center of Chiba University, Japan) under strain number IFM 63626, ITS sequence was deposited in GenBank under accession number KT808269. The molecular investigation confirmed the mycological diagnosis and histopathological data led to the final diagnosis of chronic cutaneous granulomatous infection due to *Chrysosporium keratinophilum*.

**FIGURE 4:** **(A)** After incubating at 25°C for 2 weeks, colonies appeared yellowish white, fluffy, and dense, powdery at the center on potato dextrose agar (PDA). **(B)** Hyaline hyphae bearing conidia which were terminal or lateral, sessile or on short, cylindrical protrusions, thick-walled, obovoid to clavate with conspicuous basal scars (lactophenol solution, ×400).

## Discussion

The genus *Chrysosporium* contains morphologically simple fungi with one-celled, thallic conidia. With this definition, numerous unrelated species have been affiliated to the genus. Confusion has particularly been caused by reporting species of *Emmonsia* in the Onygenalean family *Ajellomycetaceae* comprising pulmonary colonizers of wild rodents, under the name *Chrysosporium* (Hubalek et al., 1998). In contrast, *Chrysosporium* species according to the current definition either reside as saprobes in habitats enriched with keratin such as bird feathers and animal hair when related to *Onygenaceae* (De Hoog et al., 2000; Hubalek, 2000), or cause skin infections in reptiles when affiliated to *Nannizziopsiacea* (Stchigel et al., 2013). In many reports in the literature, the etiologic agent had been identified only at genus level, which obviously is non-informative (Levy et al., 1991).

*Chrysosporium keratinophilum* is the anamorph of *Aphanoascus keratinophilus*, which is a member of *Onygenaceae* (Vidal et al., 2000). Species in this family are environmental saprobes on keratinous debris (Vidal et al., 2000). Asymptomatic carriage by animals and sometimes humans has been described (Woodgyer, 1977). Some species may be involved in human superficial infection and onychomycosis at low levels of virulence (Hocquette et al., 2005). Deep infections are extremely rare in immunocompromised patients (Warwick et al., 1991). In a retrospective study of onychomycosis in humans with diabetes mellitus, *C. keratinophilum* was isolated in 2.9% of the cases (Manzano-Gayosso et al., 2008). This suggests an advantage for the fungus with metabolic or immune disorders of the host. Our case concerned an exceptionally severe infection in an apparently immunocompetent female. Recent studies of primary immunodeficiencies (PIDs), a group of hereditary immune disorders with increased susceptibility to infection, have led to significant breakthroughs in our understanding of cellular and molecular mechanisms that predispose to both invasive and mucocutaneous fungal infections. Given the severity of the case, the recurrence of the fungus over decades, and the occurrence of similar infections in family members, a rare inherited immune disorder such as homozygous mutations in the CARD9 gene involved in the C-type lectin pathway may be surmised (Alves de Medeiros et al., 2016; Wang and van de Veerdonk, 2016). Unfortunately, our patient was lost for follow-up before this was realized.

Etiology of *C. keratinophilum* in our case was proven by histological examination and mycological examination with presence of identical hyphal elements in both clinical specimens from neck and trunk. And two times of tissue biopsy culture revealed the same agent. These data provided strong evidence in favor of its pathogenicity in this exceptional, subcutaneous granulomatous infection. ITS sequencing further confirmed that the same species, which is not part of the commensal fungal flora of human skin, was involved in all lesions. The scaling lesions spontaneously appearing on the patient’s trunk for over several decades caused by *C. keratinophilum* were prior to the neck lesions, which suggests fungal infection on the neck might have been acquired by scratching. The nodular lesions remind one of chromoblastomycosis because of significant dermal acanthosis, but differs by presence of exudates and septate hyphal elements rather than muriform cells in tissue. *In vivo* studies have shown the ability of *C. keratinophilum* to induce granulomatous lesions in white mice (Otcenasek and Dvorak, 1964; Hubalek and Hornich, 1977). However, to our knowledge, the species has never been reported from a cutaneous granulomatous infection in humans. Remarkably, the neck lesions took a different clinical aspect during pregnancy, strongly suggesting a hormonal contribution in addition to the surmised immune disorder. Similar aggravation of the infection during pregnancy was reported, e.g., *Veronaea botryosa* (Bonifaz et al., 2013) and *Exophiala spinifera* (Bonifaz et al., 2013; Wang et al., 2013). However, it remains unexplained why the trunk lesions remained as mildly hyperkeratotic patches during the same period of pregnancy. At present, no standard antifungal therapy can be recommended for *Chrysosporium* infections. In this case, the patient showed satisfactory response to the treatment with itraconazole, although she discontinued the follow-up. Considering the chronic course of the infection and the risk of sudden expansion and aggravation under hormonal influence, adequate monitoring to timely adjust the therapeutic regimen is recommended.

## Ethics Statement

The study was carried out in accordance with the Declaration of Helsinki and was approved by the Committee on Ethics of Biomedical Research, Second Military Medical University (Shanghai, China). The written informed consent was obtained from the study patient.

## Author Contributions

JM, BP, SH, YH, TM, YY, YL, PA, WP, DD, YG, PZ, WL, and SD contributed to the conception of the work, the acquisition, analysis and interpretation of the clinical features and fungal characteristics. SH, JM, BP, WL, and SD substantially contributed to drafting and critically revising the work. All authors read and approved the final manuscript.

## Conflict of Interest Statement

The authors alone are responsible for the content and writing of the paper. The authors declare that the research was conducted in the absence of any commercial or financial relationships that could be construed as a potential conflict of interest.

## References

[B1] Alves de MedeirosA. K.LodewickE.BogaertD. J.HaerynckF.Van DaeleS.LambrechtB. (2016). Chronic and invasive fungal infections in a family with CARD9 deficiency. *J. Clin. Immunol.* 36 204–209. 10.1007/s10875-016-0255-826961233

[B2] BonifazA.DavoudiM. M.de HoogG. S.Padilla-DesgarennesC.Vazquez-GonzalezD.NavarreteG. (2013). Severe disseminated phaeohyphomycosis in an immunocompetent patient caused by *Veronaea botryosa*. *Mycopathologia* 175 497–503. 10.1007/s11046-013-9632-523471534

[B3] De HoogG. S.GuarroJ.FiguerasM. J.GenéJ.HubalekZ. (2000). *Atlas of Clinical Fungi* 2nd Edn Spain: Reus.

[B4] HocquetteA.GrondinM.BertoutS.MalliéM. (2005). *Acremonium, Beauveria, Chrysosporium, Fusarium*, Onychocola, *Paecilomyces, Penicillium, Scedosporium* and *Scopulariopsis* fungi responsible for hyalohyphomycosis. *J. Mycol. Méd.* 15 136–149.

[B5] HubalekZ. (2000). Keratinophilic fungi associated with free-living mammals and birds: revista iberoamericana de micologia. *Rev. Iberoam. Micol.* 17 93–103.15762800

[B6] HubalekZ.HornichM. (1977). Experimental infection of white mouse with *Chrysosporium* and *Paecilomyces*. *Mycopathologia* 62 173–178. 10.1007/BF00444111563979

[B7] HubalekZ.NesvadbovaJ.HalouzkaJ. (1998). Emmonsiosis of rodents in an agroecosystem. *Med. Mycol.* 36 387–390. 10.1111/j.1365-280X.1998.00177.x10206748

[B8] LevyF. E.LarsonJ. T.GeorgeE.MaiselR. H. (1991). Invasive *Chrysosporium* infection of the nose and paranasal sinuses in an immunocompromised host. *Otolaryngol. Head Neck Surg.* 104 384–388. 10.1177/0194599891104003171902943

[B9] Manzano-GayossoP.Hernandez-HernandezF.Mendez-TovarL. J.Palacios-MoralesY.Cordova-MartinezE.Bazan-MoraE. (2008). Onychomycosis incidence in type 2 diabetes mellitus patients. *Mycopathologia* 166 41–45. 10.1007/s11046-008-9112-518373212

[B10] OtcenasekM.DvorakJ. (1964). The isolation of *Chrysosporium keratinophilum* (Frey) carmichael 1962 and similar fungi from czechoslovakian soil. *Mycopathol. Mycol. Appl.* 23 121–124. 10.1007/BF0204926714205727

[B11] StchigelA. M.SuttonD. A.Cano-LiraJ. F.CabanesF. J.AbarcaL.TintelnotK. (2013). Phylogeny of chrysosporia infecting reptiles: proposal of the new family *Nannizziopsiaceae* and five new species. *Persoonia* 31 86–100. 10.3767/003158513X66969824761037PMC3904055

[B12] VidalP.VinuesaM. A.Sanchez-PuellesJ. A.GuarroJ. (2000). “Phylogeny of the anamorphic genus Chrysosporium and related taxa based on rDNA internal transcribed spacer sequences,” in *Biology of Dermatophytes and other Keratinophilic fungi* eds KushwahaR. K. S.GuarroJ. (Spain: Bilbao) 22–28.

[B13] WangL.SheX.LvG.ShenY.CaiQ.ZengR. (2013). Cutaneous and mucosal phaeohyphomycosis caused by *Exophiala spinifera* in a pregnant patient: case report and literature review. *Mycopathologia* 175 331–338. 10.1007/s11046-012-9611-223334555

[B14] WangX.van de VeerdonkF. L. (2016). When the fight against fungi goes wrong. *PLoS Pathog.* 12:e1005400 10.1371/journal.ppat.1005400PMC474206226845151

[B15] WarwickA.FerrieriP.BurkeB.BlazarB. R. (1991). Presumptive invasive Chrysosporium infection in a bone marrow transplant recipient. *Bone Marrow Transplant.* 8 319–322.1756331

[B16] WoodgyerA. J. (1977). Asymptomatic carriage of dermatophytes by cats. *N. Z. Vet. J.* 25 67–69. 10.1080/00480169.1977.34360275693

